# Secure Clustering Strategy Based on Improved Particle Swarm Optimization Algorithm in Internet of Things

**DOI:** 10.1155/2022/7380849

**Published:** 2022-07-16

**Authors:** Zhanbiao Bao

**Affiliations:** Center of Education Technology, Henan University of Economics and Law, Zhengzhou, Henan 450046, China

## Abstract

This paper proposes a secure clustering strategy based on improved particle swarm optimization (PSO) in the environment of the Internet of Things (IoT). First, in the process of cluster head election, by considering the residual energy and load balance of nodes, a new fitness function is established to evaluate and select better candidate cluster head nodes. Second, the optimized adaptive learning factor is used to adjust the location update speed of candidate cluster head nodes, expand the local search, and accelerate the convergence speed of global search. Finally, in the stage of forwarding node election and data transmission, in order to reduce the energy consumption of forwarding nodes, each cluster head node elects a forwarding node among the ordinary nodes in its cluster, so that the elected forwarding nodes have the optimal energy and location relationship. Experiments show that the proposed method effectively prolongs the network lifetime compared with the comparison methods. The average node degree of the proposed method is less than 2.5.

## 1. Introduction

With the development of information society, the information industry is more and more vigorous, and the scope of information application is more and more extensive [1]. Especially in the process of the big data era, the acquisition of information has attracted more and more attention, and become one of the important hotspots of scientific research and value-added industry [2–4]. Effective information acquisition is the basis of information transmission, processing, mining, and application. Sensors connect the physical world and the digital world by capturing and revealing the physical phenomena of the world and transforming them [5]. Wireless sensor network (WSN) is a self-organized network composed of a large number of sensor nodes with information collection, processing, and transmission functions. Each sensor node can realize the data collection, processing, and transmission of the sensing area, and the whole network can cooperate to complete the information collection in the target area [6–8]. Through the deployment and use of the network, the ability of human society to obtain information can be enhanced. It has changed the situation that people only rely on their own feelings and simple tools to perceive information since ancient times and greatly improved the accuracy and sensitivity of human access to data and information [9, 10].

WSN is often used to monitor events of interest in the surrounding environment. A typical WSN monitoring system consists of sensor nodes, base stations, and monitoring centers [11–13]. The remote user or monitoring center can send data acquisition, processing, and transmission commands to the sensor nodes in the network through the base station, and finally, receive the interested data through the base station [14–16].

In the environment of IoT, aiming at the problems of large node energy consumption and short network life cycle caused by the unbalanced location distribution of cluster head nodes screened by clustering routing protocol of wireless sensor networks and unreasonable data transmission path of forwarding nodes, a secure clustering strategy based on improved PSO algorithm in the IoT environment is proposed. The innovations of the proposed method lie in the following:

1. In the process of cluster head election, considering the residual energy and load balance of nodes, a new fitness function is established to evaluate and select better candidate cluster head nodes, which effectively shortens the communication distance.
2. The optimized adaptive learning factor is used to adjust the position update speed of candidate cluster head nodes, and the concave function nonlinear decreasing strategy is used to improve the inertia weight, which speeds up the convergence speed of global search.
3. For each cluster head node, a forwarding node is selected from the ordinary nodes in its cluster, so that the selected forwarding node has the optimal energy and location relationship, and the node communication overhead is reduced.

The remaining chapters of this paper are arranged as follows.  Section 2 introduces the related research in this field; Section 3 introduces the system model; Section 4 introduces the proposed clustering routing algorithm based on improved PSO algorithm; Section 5 is the experiment, and Section 6 summarizes this study.

## 2. Related Works

Compared with plane routing, cluster routing saves the energy consumption of the network to the greatest extent, facilitates data fusion, and is easier to expand [17–19]. As a simple and effective random search algorithm, intelligent algorithm has good application prospects in finding the optimal solution of function and neural network recognition [20]. In the late 19th century, James Kennedy of the United States proposed PSO for the first time. It is famous for its simplicity and effectiveness. Therefore, scholars at home and abroad choose PSO algorithm in cluster head selection. Reference [21] defined a new cost function to minimize the communication distance between cluster members and cluster heads and used the PSO to select cluster heads with higher energy to optimize network clustering. Reference [22] proposed a new clustering mode EECS for wireless sensor networks, which specified the size of clusters in the network. Clusters far from the base station have a larger radius, and clusters close to the base station have a smaller radius, so as to balance the energy consumption of cluster heads. Reference [23] proposed a new hierarchical clustering protocol PSO-HC, which balanced the network energy consumption by reducing the number of cluster heads and transmitted the information collected by cluster heads to the base station by multihop. Based on the clustering of the LEACH protocol, reference [24] used the ant colony algorithm to optimize the distance location between each node and the base station and obtained the best path. Through this path, the cluster head transmitted the information to the next cluster head in sequence until the information was transmitted to the base station.

Reference [25] proposed an improved PSO algorithm to optimize the running time of the network. The algorithm comprehensively considered the factors of energy and distance to realize the selection of target nodes and proposed the introduction of relay nodes to share the transmission work of cluster head nodes. Reference [26] combined harmony search (HS) algorithm and PSO to select cluster head nodes. The algorithm not only had the efficient search efficiency of harmony search algorithm but also had the dynamic ability of the PSO algorithm, which could better improve the performance of the network. According to the uneven clustering algorithm, reference [27] used ant colony optimization algorithm to calculate the optimal distance between the node and the base station and transmitted the data of each cluster head node to the base station through the selected optimal path. The disadvantage of this algorithm is that the path from each cluster head to the base station needs to be calculated, so it will lead to excessive energy consumption. Reference [28] proposed a clustering strategy based on FBECS (fuzzy based enhanced cluster head selection). In the clustering stage, fuzzy logic algorithm was used to calculate the qualification index of each node according to the residual energy of the node and the distance between the node density and the base station. The node generated the cluster head by comparing the randomly generated random number with the qualification index. Reference [29] proposed a clustering method based on energy center search using PSO (EC-PSO), which used geometric method to select CHs and searched energy centers in CHs selection.

## 3. System Model

### 3.1. Network Model

In order to better optimize the algorithm, this model makes the following assumptions.

1. The nodes are randomly deployed in the target area. After deployment, the nodes will no longer move, and each node has a unique ID.
2. All nodes have the same initial energy, computing power, and communication ability and can automatically adjust the transmission power.
3. Each node can communicate with the base station independently, and the location of the base station is known.
4. The node can calculate its relative position according to the angle of arrival and signal strength.

### 3.2. Energy Model

The same energy model as LEACH is used for communication between nodes. According to the distance $d_{ij}=\sqrt{{\left(x_{i}-x_{j}\right)}^{2}+{\left(y_{i}-y_{j}\right)}^{2}}$ between node *i* and node *j*, the channel model is selected. The energy consumed by a node to send *k* bit data to the node with a distance of d is

(1) $$\begin{array}{c} E_{TX}\left(k,d\right)\left\{\begin{array}{c} k\left(E_{\text{elec}}+\alpha_{fs}d^{2}\right),d<d_{0},\\ k\left(E_{\text{elec}}+\alpha_{mp}d^{2}\right),d>d_{0}, \end{array}\right.\\ d_{0}=\sqrt{\frac{\alpha_{fs}}{\alpha_{mp}}}. \end{array}$$

The energy consumed by the node to receive and fuse *k* bit data is

(2) $$\begin{array}{c} E_{RX}\left(k\right)=kE_{elec},\\ E_{DA}\left(k\right)=kE_{da}, \end{array}$$

where *E*_elec_ is the energy consumed to receive or send 1 bit data and *E*_*da*_ is the energy consumed by the node to fuse 1 bit data. The transmission model selected by the node for communication is determined by d_0_. *α*_*fs*_ and *α*_*mp*_ are the energy required for power amplification of free space channel model and multipath fading model. When the distance between nodes d < d_0_, choose the free space channel model; otherwise, choose the multipath fading model.

## 4. Clustering Routing Algorithm Based on Improved PSO Algorithm

### 4.1. Cluster Head Election

#### 4.1.1. Cluster Head Initialization

Because the calculation of the PSO algorithm is relatively complex, in order to avoid increasing the energy consumption of nodes in election calculation, the clustering and routing calculation based on the PSO algorithm will be completed by the base station with unlimited energy. In the initialization process, all nodes send their residual energy, location, and number information to the base station, and the base station receives and saves the information of each node. After the base station completes the clustering calculation based on the PSO algorithm, the base station broadcasts the calculation results. Each surviving node obtains the specific location information of the elected node and routing node according to the received broadcast information. PSO algorithm selects particles randomly, which is easy to fall into local optimization, resulting in uneven distribution of nodes in the cluster. To solve this problem, the energy of nodes participating in cluster head node election is limited.

Suppose there is *N* surviving nodes in the WSN, the energy of node *i* is *E*(*i*), and the base station calculates the average residual energy of all nodes in the WSN as *E*_*a*_=1/*N*∑_*i*=1_^*N*^*E*(*i*).

In order to ensure that the selected cluster head nodes have sufficient energy to process the data in the cluster, the base station forms a set EA of all nodes with energy greater than or equal to *E*_*a*_, then randomly selects *K* nodes from the EA, and stores them in the candidate cluster head node set to form a particle. After initially determining a group of candidate cluster head nodes, other noncluster head nodes join the cluster head nodes closest to them, respectively, to complete the establishment of initial clustering. Then, continue to select *K* nodes in EA in a random way, conduct a total of *M* times of screening, and finally generate the *M* groups of initial cluster head node set; that is, *M* particles, and form the *M* groups of clusters.

#### 4.1.2. Fitness Function

The cluster head node is responsible for most activities and needs to consume more energy, which may lead to premature failure due to excessive energy consumption and reduce the performance of the whole network. Therefore, when selecting the cluster head node, it should consider the following two aspects: select the cluster head node with large residual energy and balance the load of the cluster head node at the same time.

First, consider selecting the cluster head node set with large residual total energy. Suppose that *K* is the number of cluster head nodes selected by the current particle. *CH* represents the cluster head set and *CH*_*k*_ represents the cluster head node of *k* cluster. The ratio *f*_1_ of the current residual energy of all nodes to the residual energy of the cluster head node set is

(3) $$\begin{array}{c} f_{1}=\frac{\sum_{i=1}^{N}E\left(i\right)}{\sum_{i=1}^{N}E\left(CH_{k}\right)}, \end{array}$$

where *E*(*i*) represents the residual energy of the sensor node *i* in the particle.

After the current particle selects the cluster head node, the set *CS*_*k*_ is used to represent the member node set of the cluster *k*. *C*_*k*_ is used to count the number of member nodes in the cluster *k*. If the node *j* joins the cluster *k*, it can be expressed as *j* ∈ *CS*_*k*_, and the *C*_*k*_ plus 1.

After clustering the current particles, it should further consider the load of the current cluster. The load of the cluster mainly includes the load in the cluster and the load between clusters. For the load balancing in the cluster, it is considered from two aspects: the number of member nodes in the cluster and the distance from the member nodes in the cluster to the cluster head.

Let *f*_2_ represent the average of the deviation between *s* and the maximum distance between each cluster head node and its nodes in the cluster.

(4) $$\begin{array}{c} f_{2}=\sum_{k=1}^{K}\frac{1}{K}\left|\max\left(\sum_{j=1}^{N}\text{d}\left(j,CH_{k}\right)-s\right)\right|. \end{array}$$

Let *f*_3_ represent the difference between the number of member nodes in each cluster and the average number of members in the cluster. The smaller the difference, the closer the number of members between clusters, and the more effective it is to balance the energy consumption between cluster heads, so as to prolong the life cycle of the network:

(5) $$\begin{array}{c} f_{3}=\sum_{k=1}^{K}\frac{1}{K}\left|\frac{N}{C_{k}}-K\right|, \end{array}$$

where d(*x*, *y*) refers to the distance between node *x* and node *y*. *r* is the radius of clusters when the whole network area can be covered. Ideally, the area of each cluster is evenly distributed in the network area, and there is no coverage area between each cluster. The area of each cluster should be *A*/(pro × *N*), where *A* is the area of the whole network area, *pro* is the preset proportion of cluster heads and pro × *N* is the number of cluster heads, so the ideal *r* value is $\sqrt{A/\left(\text{pro}\times N\right)}$.

*f*_4_ represents the average distance between cluster heads. The smaller the average distance between cluster heads, the smaller the load between clusters, which can reduce the communication energy consumption of the network.

(6) $$\begin{array}{c} f_{4}=\frac{2\left.\left(\sum_{k=1}^{K-1}\sum_{j=k+1}^{K}d\left(CH_{k},CH_{j}\right)\right)\right)}{\left(\left(K-1\right)/K\right)}. \end{array}$$

In the fitness function, the node residual energy and load balance are comprehensively considered, and the multiobjective optimization problem is transformed into a single objective optimization problem by means of weighted sum:

(7) $$\begin{array}{c} F=\alpha f_{1}+\beta f_{2}+\chi f_{3}+\delta f_{4}, \end{array}$$

where *α*, *β*, *χ*, and *δ* are weighting factors.

#### 4.1.3. Update Method of Speed and Position

According to the initial fitness calculation and the initially generated local optimal location and global optimal location, start a round of iterative calculation. First, update the location of the candidate cluster head node set, and then calculate the fitness of the candidate cluster head node after location update. In order to complete the location update of the candidate cluster head node set and obtain the optimization results, let the velocity components of the candidate cluster head nodes in the *x* and *y* directions be *v*_*x*_ and *v*_*y*_, respectively, and the position components be *x*_*x*_ and *x*_*y*_, respectively.

The calculation of the two velocity components is initially generated randomly, but in each subsequent iteration, it is determined according to the change relationship between the velocity component of the previous round of the candidate cluster head node set and the local optimal position (*p*_*xi*_, *p*_*yi*_) and the global optimal position (*p*_*xg*_, *p*_*yg*_). The specific calculation is as follows:

(8) $$\begin{array}{c} \left\{\begin{array}{c} v_{x}\left(t\right)=wv_{x}\left(t-1\right)+c_{1}l_{1}\left(p_{xi}\left(t-1\right)-x_{xi}\left(t-1\right)\right),\\ +c_{2}l_{2}\left(p_{xg}\left(t-1\right)-x_{xi}\left(t-1\right)\right),\\ v_{y}\left(t\right)=wv_{y}\left(t-1\right)+c_{1}l_{1}\left(p_{yi}\left(t-1\right)-x_{yi}\left(t-1\right)\right),\\ +c_{2}l_{2}\left(p_{yg}\left(t-1\right)-x_{yi}\left(t-1\right)\right), \end{array}\right. \end{array}$$

where *w* is the inertia weight, which indicates the influence of the speed of the previous *t* − 1 iteration of the candidate cluster head node set on the speed of the candidate cluster head node set in this *t* iteration. *c*_1_ is a cognitive learning factor and *c*_2_ is a social learning factor, which, respectively, represent the acceleration weight of the candidate cluster head node set close to the local optimal position and the global optimal position. *l*_1_, *l*_2_ ∈ (0,1) are the random numbers.

Based on the two velocity components, the calculation method of the position components *x*_*xi*_(*t*) and *x*_*yi*_(*t*) of the candidate cluster head node in the direction *x* and *y* is as follows:

(9) $$\begin{array}{c} x_{xi}\left(t\right)=x_{xi}\left(t-1\right)+v_{xi}\left(t\right),\\ x_{yi}\left(t\right)=x_{yi}\left(t-1\right)+v_{yi}\left(t\right). \end{array}$$

#### 4.1.4. Improved Inertia Weight

Among the parameters that can be adjusted by the PSO algorithm, researchers often improve the important parameter of inertia weight. A larger inertia weight value is conducive to improve the global search ability of the PSO algorithm, and a smaller weight value will enhance the motion ability of particles.

Under the same convergence accuracy, the concave function decreasing strategy greatly improves the convergence speed of PSO compared with other improved strategies, and can more effectively control the balance between global search and local search.

The rule for improving inertia weight by using concave function nonlinear decreasing strategy is as follows:

(10) $$\begin{array}{c} w=\left(w_{\max}-w_{\min}\right)\left[\left(\frac{C_{\text{Cur}}}{C_{\text{Loop}}}\right)2+2\frac{C_{\text{Cur}}}{C_{\text{Loop}}}\right]+w_{\text{max}}, \end{array}$$

where *w* ∈ [0.5, 0.9] and *C*_Cur_ represent the number of rounds of the current iteration and *C*_Loop_ represents the total number of iterations.

#### 4.1.5. Location Mapping Strategy

After each round of iteration, the location of the candidate cluster head node set will be updated, and the updated node location may not find a matching surviving node in the WSN. At this time, location mapping is needed. The basic idea is to adopt the proximity principle to map the updated location to the location of the nearest surviving node. Take *x*_*xi*_ and *x*_*yi*_ as the updated node coordinates and *CM*_*nx*_ and *CM*_*ny*_ as the coordinates of the surviving node *CM*_*n*_ in the network. The location mapping process is as follows:

(11) $$\begin{array}{c} CM_{n}=\left\{\left(CM_{nx},CM_{ny}\right)|\text{min}\sqrt{{\left(CM_{nx}-x_{xi}\right)}^{2}+{\left(CM_{ny}-x_{yi}\right)}^{2}}\right\}. \end{array}$$

The location mapping strategy solves the mismatch between the updated location and the actual surviving node location caused by the discrete distribution of network nodes. When the updated position coordinates of multiple nodes are the same, it is necessary to set a flag while updating the node. When updating and mapping the positions of other nodes, first check whether the flag has been identified as the cluster head node. If so, select the next closest node position in turn for mapping.

After completing the location mapping, take the candidate cluster head node set after the location update as the optimization result, and calculate the fitness value of each candidate cluster head node set. According to the calculation results, the local optimal location of each group of candidate cluster head node set and the global optimal location of *M* groups of cluster head node sets in this round are updated. If the iteration is not finished, continue to update and map the location of candidate cluster head nodes. Otherwise, the candidate cluster head node set of the global optimal position is calculated as the optimal cluster head node set, and the cluster head election is completed.

After completing the cluster head election, the base station further calculates the distance from the noncluster head node to each cluster head node and adds the noncluster head node to the nearest cluster head node to complete clustering. Ordinary nodes only send data. After receiving the data from ordinary nodes, the cluster head node performs data fusion and then sends it to the corresponding forwarding node. The forwarding node needs to be further selected from ordinary nodes. It receives the data from the cluster head, selects the optimal path to the base station, and sends the data to the base station.

### 4.2. Election and Data Transmission of Forwarding Nodes

#### 4.2.1. Election of Forwarding Nodes

After the cluster head node election is completed, the corresponding forwarding node will be selected for the cluster head node. If there are too few forwarding nodes in the network, multiple cluster head nodes send data to the base station through a small number of forwarding nodes, which will increase the energy consumption of forwarding nodes. To solve this problem, the existing WSN routing protocol adopts the way that one cluster head node corresponds to one forwarding node to increase the number of forwarding nodes, but it selects all nodes randomly without considering whether the residual energy and location of the selected nodes are balanced.

In the forwarding node election, the improved PSO algorithm of the above cluster head node election is adopted to elect a forwarding node for each cluster head node among the ordinary nodes in its cluster, so that the elected forwarding node has the optimal energy and location relationship, and avoid speeding up its energy consumption due to too few forwarding nodes in WSN. In the calculation and evaluation of forwarding nodes, because forwarding nodes can only be elected in one cluster, the calculation methods of energy factor and location balance factor are different from those of cluster head node election. Similarly, *N* represents the number of surviving nodes in the WSN. After selecting *K* cluster head nodes, the WSN is divided into *K* clusters. During initialization, according to the cluster head node screening method, candidate forwarding nodes with high residual energy are screened out in each cluster to form a set of candidate forwarding nodes. Each candidate set contains *K* nodes. After initialization, the number of ordinary nodes is *N* − 2*K*. Let *E*_*RN*_^*r*^(*i*) represent the residual energy of candidate forwarding node *RN*_*i*_ in round *r*, and *E*_*CN*_^*r*^(*i*) represent the residual energy of ordinary node *CN*_*j*_ in round *r*. The calculation formula of energy factor fit_1_ is

(12) $$\begin{array}{c} {\text{fit}}_{1}=\frac{\left(N-2K\right)\sum_{j=1}^{N-2K}E_{RN}^{r}\left(i\right)}{K\sum_{j=1}^{N-2K}E_{CN}^{r}\left(i\right)}. \end{array}$$

Let d(*CN*_*k*_, *CH*_*j*_) represent the distance between the ordinary node *CN*_*k*_ and the corresponding cluster head node *CH*_*j*_, d(*RN*_*i*_, *BS*) represent the distance between the forwarding node *RN*_*i*_ and the base station *BS*, d(*RN*_*i*_, *CH*_*j*_) represent the distance between the forwarding node *RN*_*i*_ and the corresponding cluster head node *CH*_*j*_, and d(*RN*_*i*_, *RN*_*m*_) represent the distance between the forwarding nodes *RN*_*i*_ and *RN*_*m*_. The calculation method of the location equalization factor fit_2_ of the forwarding node is as follows:

(13) $$\begin{array}{c} {\text{fit}}_{2}=\frac{K^{2}\sum_{j=1}^{N-2K}d\left(CN_{k},CH_{j}\right)}{\left(N-2K\right)\left(\sum_{i=1}^{K}\text{d}\left(RN_{i},BS\right)+\sum_{i=1}^{K}\text{d}\left(RN_{i},CH_{j}\right)+\sum_{i=1}^{K-1}\sum_{m=i+1}^{K}d\left(RN_{i},RN_{m}\right)\right)}, \end{array}$$

where the ordinary node *CN*_*k*_ is located in the cluster where the cluster head node *CN*_*k*_ is located and the candidate forwarding node *RN*_*i*_ corresponds to the cluster head node *CH*_*j*_. The closer the candidate forwarding node set is to the base station, the smaller the distance between the cluster head node and the forwarding node in each cluster; the smaller the distance between the forwarding nodes in the candidate forwarding node set, the more balanced the location distribution of the candidate forwarding node set, and the greater the fit_2_ value.

Based on the ability factor and location balance factor of candidate forwarding node election, the fitness function F2 for the evaluation of candidate forwarding node set constructed by weighting method is as follows:

(14) $$\begin{array}{c} F_{2}=b{\text{fit}}_{2}+\left(1-b\right){\text{fit}}_{2}, \end{array}$$

where *b* ∈ (0,1] is the weight. The higher the residual energy of the candidate forwarding node set and the more balanced the location, the greater the fitness value of the candidate forwarding node set, indicating that the candidate forwarding node set is better. In the iterative election process of candidate forwarding node set, the speed update and location mapping method similar to cluster head node election is used to select the optimal forwarding node set.

#### 4.2.2. Data Transmission

WSN forward routing mainly selects relay nodes for cluster heads far away from the base station, and relay nodes reduce the load of cluster heads by forwarding data packets from cluster heads. Assuming that the data packet needs to be sent to the base station through *n* hop; that is, through *n* − 1 relay nodes, the optimal relay node should have the following characteristics:

1. The distance between relay nodes should be as balanced as possible.
2. The relay node should have high energy to meet the data transmission requirements.
3. The total distance should be as close as possible to the direct communication distance between the cluster head and the base station.
4. The selection of relay nodes should avoid selecting other cluster heads.
5. The load of relay nodes should be as small as possible to avoid over development.

According to the above requirements, the corresponding fitness function is designed, which can be expressed as

(15) $$\begin{array}{c} F_{3}=\varepsilon \left(\frac{E_{\text{min}}}{E_{\text{init}}}+\frac{1}{{\text{load}}_{\max}}\right)+\phi \left(\frac{{\text{d}}_{\min}}{{\text{d}}_{\max}}+\frac{{\text{d}}_{\text{init}}}{{\text{d}}_{\text{total}}}\right), \end{array}$$

where *E*_min_ is the node with the smallest energy among the relay nodes; the load of the node is determined by the number of data packets received by the node. load_max_ is the node with the largest load in the relay nodes; d_min_ and d_max_ are the minimum and maximum distance between adjacent nodes in the forward routing path, respectively; d_init_ and d_total_ are the sum of the distance between the cluster head and the base station and the sum of distance of the whole forward routing path; *ε*=0.5+0.5*E*_loss_/*E*_total_; *ϕ*=1 − *ε*. The total energy consumption of the nodes in the cluster is changed into the energy consumed by the cluster head that needs to plan the route, and the total energy in the cluster is changed into the initial energy of the cluster head. With the operation of the network, the parameter weight ratio is dynamically adjusted.

## 5. Experiments and Analysis

### 5.1. Experimental Setup

Simulating the generation of WSN in MATLAB and setting the base station outside the network, in this environment, the secure clustering strategy based on improved PSO algorithm is tested. The experimental computer is configured with 2.3 GHz, Intel Core I7, 8 GB RAM, and 64 bit Windows10. The experimental environment and parameter settings related to WSN initialization, cluster head node, forwarding node election, and data processing are shown in Table 1.

### 5.2. Performance Index Comparison of Topology Generated by Different Schemes

In order to prove the performance of the proposed method under the same experimental conditions, the proposed method is compared with the methods in references [28, 29], and the comparison results are shown in Figure 1. In order to compare the algorithms effectively without losing generality, it is assumed that *n* sensor nodes are randomly deployed in the target monitoring area of 200 × 200.

As can be seen from Figure 1(a), the average link length of the three methods continues to decrease with the growth of *n*. The proposed method can maintain the global connectivity of the network with a short average link length and has strong advantages in reducing the overall energy consumption of the network.

Figure 1(b) shows the comparison results of the average node degree of the three control schemes. It can be seen from the figure that the average node degree of the other two methods tends to rise with the increase of the network scale, while the topology obtained by the proposed method has a low average node degree, which is basically maintained below 2.5, and the average node degree is relatively stable and will not change greatly with the change of the network scale. It shows that this method has good stability and low interference.

As can be seen from Figure 1(c), when the network size is 70, the average number of joint points of the methods in references [28, 29] is 3.0 and 2.3, respectively, and the number of joint points of the proposed method is 0. The number of joint points of the methods in references [28, 29] decreases with the continuous growth of the network size, but the method in this paper has better stability and can ensure that there are basically no joint points under different network sizes. This is because the proposed method comprehensively considers the residual energy and load balance of nodes, establishes a new fitness function, and can select better candidate cluster head nodes. Therefore, compared with the other two methods, the proposed method can better ensure the connectivity of topology when clusters are connected.

### 5.3. Location Balance Test of Cluster Head Nodes

The location balance factor reflects the distribution balance of cluster head node set and forwarding node set in WSN. The more balanced the node distribution is, the smaller the total communication distance in WSN communication is, and the lower the node energy consumption will be. Based on the above experimental environment, the total distance from all ordinary nodes to cluster heads and the total distance from all cluster head nodes to base stations in multiple iterations of the methods proposed in this paper, references [28, 29] are tested, respectively. The experimental results are shown in Figures 2 and 3, respectively.

As can be seen from Figures 2 and 3, with the increase of the number of iterations, the total distance from all ordinary nodes to cluster heads and the total distance from all cluster heads to base stations in the three methods become smaller and smaller. In the method of reference [28], the energy and location of nodes are not considered in cluster head election. Initially, the two distances in Figures 2 and 3 are the largest, but the two distances drop rapidly after 2600 rounds. This is because their communication distance is large, energy consumption is large and unbalanced, and node death is fast. With the large reduction of surviving nodes, their communication distance decreases, and the life cycle of WSN is greatly shortened. This is because, the proposed method elects a forwarding node for each cluster head node among the ordinary nodes in its cluster so that the selected forwarding node has the optimal energy and location relationship, which effectively reduces and balances the node energy consumption. The number of dead nodes decreases linearly and slowly, the change is relatively stable and prolongs the life cycle of WSN.

The method in reference [29] considers the location information. At the beginning, the two distances are relatively reduced, the energy consumption is reduced, and the life cycle of WSN is prolonged. The optimization of the inertia weight in the method of reference [29] makes the elected cluster head nodes close to the global optimization. The two distances measured at the beginning are lower than those in the method of reference [28], the node energy consumption is reduced, and the life cycle of WSN is longer than that in the method of reference [28]. The methods in references [28, 29] have fewer surviving nodes due to the proliferation of dead nodes in the later stage of iteration. The measured two distances are smaller than the proposed method, but the life cycle is smaller.

## 6. Conclusion

A secure clustering strategy based on improved PSO algorithm in the environment of IoT is proposed. Considering the residual energy and load balance of nodes, a new fitness function is established, the better candidate cluster head nodes are evaluated and selected. The location update speed of candidate cluster head nodes is adjusted through the optimized adaptive learning factor, so as to elect a forwarding node for each cluster head node among the ordinary nodes in its cluster for reducing the energy consumption of forwarding nodes. Experiments show that under the same conditions, the average node degree of the proposed method is less than 2.5, which is better than the comparison methods. Compared with the comparison methods, the proposed method can significantly improve the network life cycle of clustering method and optimize node energy consumption.

In WSN clustering routing protocol, the selected cluster head nodes usually accounts for only a small part of the total nodes, so it has sparse characteristics. In future research work, sparse theory can be introduced to solve the problem of cluster head node selection in WSN clustering routing. In addition, in practical applications, the location of sensor nodes is not fixed, so energy optimization can be studied for large-scale dynamic networks.

## Figures and Tables

**Figure 1:** Comparison of performance indices of topologies generated by different schemes: (a) comparison of average link length; (b) comparison of average node degree; (c) comparison of average number of joints.

**Figure 2:** Sum of distances from ordinary nodes to cluster heads in different methods.

**Figure 3:** Sum of distances between cluster heads and base station in different methods.

**Table 1:** Experimental parameters setting.

Parameter name	Value
Number of nodes	150
Base station location	(50,100)
Network scale	200 m × 200 m
*E*_fs_ (pJ.(bit·m^2^)^−1^)	10
*E*_mp_ (pJ.(bit·m^4^)^−1^)	0.002
*E*_elec_ (nJ.bit^−1^)	60
*d*0 (m)	70
Maximum number of rounds	2500
The number of iterations of the algorithm	200
Optimal number of clusters	10
Number of particle	20
Data packet length/bit	5000
Control packet length/bit	100
Node initial energy *E*0 (J)	0.7

## Data Availability

The data used to support the findings of this study are included within the article.
